# Meta-analysis on the efficacy of tourniquet on ankle trauma surgery

This article has been retracted.

**DOI:** 10.1186/2047-783X-18-55

**Published:** 2013-12-10

**Authors:** Xinhua Jiang, Baoqing Yu, Wei Qu, Jiawen He

**Affiliations:** 1 Department of Orthopaedics, Shanghai Pudong Hospital, Fudan University Pudong Medical Center, No.2800 Gongwei Road, Huinan Town, Pudong, Shanghai 201399, China

**Keywords:** Tourniquet, Limb trauma, Ankle, Operation, Meta-analysis

## Abstract

**Background:**

In our study, we used meta-analysis to study the efficacy of the tourniquet on ankle trauma surgery. Postoperative infection rate, deep venous thrombosis incidence, hospital stay, and joint range of motion were studied to compare the tourniquet and non-tourniquet groups and provide certain references for clinical decision.

**Methods:**

We searched PubMed, MEDLINE, EMBASE, and the Cochrane controlled trials register for all publications about the efficacy of tourniquet published before November 2012. The quality of included studies was evaluated by two estimators. *I*^2^-test and Q-statistic were used for heterogeneity analysis. When there was heterogeneity between studies, the random effects model analysis was applied or else the fixed effects model analysis was used.

**Results:**

Three studies were included with 166 patients suffering from ankle trauma surgery. There was no statistical difference (*P* >0.05) between the tourniquet and non-tourniquet groups on operation time (mean difference (MD) −5.45, 95% confidence intervals (CI): (−13.98, 3.09)), postoperative infection rate (relative risk (RR) 1.83, 95% CI: (0.65, 5.12)), and deep venous thrombosis incidence (RR 4.13, 95% CI: (0.47, 36.17)). But statistical significances were observed on hospital stays (MD 3.17, 95% CI: (1.39, 4.95)) and joint range of motion (MD − 5.25, 95% CI: (−9.61, −0.89)).

**Conclusions:**

In general, the efficacy of the tourniquet group is comparable to that of the non-tourniquet group. The non-tourniquet group achieved greater benefits for the joint range of motion and reduced the hospital stay. However, a larger number of primary studies is still required for future evaluation of tourniquet efficacy on ankle trauma surgery.

## Background

Tourniquets are commonly used in limb trauma surgery, playing an important role in the forearm, wrist, and ankle departments [1]. The use of the tourniquet has been advocated to improve visualization in the surgical field, shorten operation time, relieve the suffering of patients, as well as minimize intraoperative blood loss [2-4], which is more safe and efficient. However, the use of the tourniquet is accompanied by many postoperative complications: bandage injuries, cuff pressure injuries, nerve injuries, pulmonary embolism, superficial wound infections [5], neurapraxia [6,7], vessel damage [8], postoperative swelling [9], postoperative pain [10,11], muscle injury [12,13], and even acute thrombosis [14] and shock [5,15]. Therefore, the use of the tourniquet still remains controversial.

Meta-analysis is an important method to find high quality evidence to analyze the efficacy of the tourniquet. A meta-analysis showed that there were fewer operative visualization difficulties for arthroscopic knee surgery with a tourniquet compared to without a tourniquet [16]. Tai et al. demonstrated that using a tourniquet in total knee arthroplasty could save time but not reduce blood loss and could lead to higher risk of thromboembolic complications [17]. Smith et al. reported a meta-analysis of the efficacy of the tourniquet on foot and ankle surgery, suggesting that pain was reduced and hospital stay was shortened after surgery without using a tourniquet [18]. Nevertheless, the outcomes of using a tourniquet on ankle trauma surgery are still not fully elucidated.

In our study, we used meta-analysis to study the efficacy of the tourniquet on ankle trauma surgery. Postoperative infection rate, deep venous thrombosis incidence, hospital stay, and joint range of motion were studied to compare the tourniquet and non-tourniquet groups and provide certain references for clinical decision.

## Methods

### Literature retrieval and search strategies

We searched PubMed, MEDLINE, EMBASE, and the Cochrane controlled trials register, and used the literature tracing method to collect interesting papers on the use of the tourniquet on ankle trauma surgery published before November 2012. We then used Google Scholar to retrieve related literature. The search strategy was based on a combination of MeSH terms: (randomized controlled trial or clinical trial) and tourniquet and ankle and surgery.

### Literature screening

The studies used in our meta-analysis should meet the following inclusion criteria: (1) primary research literature published at home and abroad; (2) experiments in the studies should be randomized clinical trials or clinical controlled trials; (3) clear launch or publication time of the study; (4) explicitly stipulated sample size; (5) explicit diagnostic criteria; (6) surgical treatment was used in the study; (7) the evaluation index included operation time, hospital stays, postoperative joint range of motion, and complications; (8) scientific data collection method; and (9) proper data analysis methods.

The study was excluded if it any of the following criteria were met: (1) studies do not provide the source of cases and control and clear number of group, studies are non-therapeutic clinical studies, animal experiments, no original documents, or no clear groups; (2) indeterminate diagnostic criteria; (3) no control group; (4) no surgical treatment; (5) unscientific data collection method; (6) wrong or no data analysis methods; (7) reviews; (8) duplicate studies; or (9) retrospective analysis.

### Quality assessment and data extraction

The double parallel extraction method was applied. Two estimators assessed literature independently as follows: (1) general information including: first authors, sources, and publication time of the literature; (2) study design of each trial; and (3) sample size, features, and therapeutic outcomes.

### Statistical analysis

Meta-analysis was carried out by RevMan 5.0. Mean difference (MD) and its 95% confidence intervals (CI) were used to represent continuous data, while relative risk (RR) and its 95% CI were used to represent dichotomous data. *I*^2^-test and Q-statistic were used for heterogeneity analysis between studies. If significant Q-statistic (*P* ≤0.05) appeared, there was heterogeneity between studies and the random effect model analysis was then applied or else the fixed effect model analysis was used (*P* >0.05).

## Results

### Features of eligible literature

A total of 131 papers relating to tourniquets using in ankle trauma surgery were collected. After checking their titles and abstracts, 46 were excluded. We then carefully screened the other 82 studies due to the factors of comments, non-randomized controlled clinical trials, or animal experiments. Finally, three studies were identified as eligible trials [19-21]. Figure 1 showed the flow diagram of study selection process. All of them were small sample tests, including 166 patients in total. The smallest sample size was 32 cases, while the largest was 80 cases (see Table 1).

**Figure 1:** Flow diagram of study selection process.

**Table 1:** General information of the three eligible studies

**Author**	**Journal**	**Surgery**	**Cases ( *n *)**		**Gender (male/female)**		**Average age (years)**		**Results in tourniquet group**
			**Tourniquet**	**Non-tourniquet**	**Tourniquet**	**Non-tourniquet**	**Tourniquet**	**Non-tourniquet**	
Konrad 2005 [19]	Clin Orthop Relat	Open reduction and internal fixation (ORIF)	26	28	10/16	11/17	42.7	41.6	More postoperative swelling and pain, less range of motion
Maffulli 1993 [20]	J Bone Joint Surg	ORIF of simple, closed fractures of the distal part of the fibula	40	40	33/7	27/11	52	50	Longer operation time, more complications, less frequency of wound infection, return to work later
Omeroglu 1997 [21]	Foot Ankle	ORIF of malleolar fractures	16	16	10/6	12/4	40	37	More pain

### Comparison of operation time between tourniquet and non-tourniquet groups

All the three trials [19-21] reported 166 patients’ operation time in total. There were 82 and 84 cases in the tourniquet and non-tourniquet groups, respectively. The random effects model was chosen when heterogeneity was observed (*P* = 0.02, *I*^2^ = 73%). Results showed there was no statistical difference between the two groups (MD −5.45, 95% CI (−13.98, 3.09)), suggesting the tourniquet group had a comparable operation time to the non-tourniquet group (see Figure 2).

**Figure 2:** Meta-analysis of patients’ operation time in the tourniquet and non-tourniquet groups.

### Comparison of hospital stays between tourniquet and non-tourniquet groups

The Forest plot for the MD between the tourniquet and non-tourniquet groups in terms of length of hospital stay is shown in Figure 3. The heterogeneity for two studies [19,20] was not significant (*P* = 0.72, *I*^2^ = 0%) and the fixed effects model was chosen. Results exhibited statistical difference between the two groups (MD 3.17, 95% CI (1.39, 4.95)), indicating tourniquets could prolong patients’ hospital stay.

**Figure 3:** Meta-analysis of hospital stays of patients in the tourniquet and non-tourniquet groups.

### Comparison of joint range of motion between tourniquet and non-tourniquet groups

Two studies [19,20] reported different ankle range of motion among 66 patients in the tourniquet group and 68 in the non-tourniquet group. Heterogeneity was not observed (*P* = 0.51, *I*^2^ = 0%), so the fixed effects model was chosen. Results showed that there was a statistical difference between the two groups (MD −5.25, 95% CI (−9.61, -0.89)) and the score was 5.25 lower in the tourniquet group than in the non-tourniquet group, indicating the use of tourniquets may reduce the joint range of motion compared to the non-tourniquet group (see Figure 4).

**Figure 4:** Meta-analysis of joint range of motion in the tourniquet and non-tourniquet groups.

### Comparison of postoperative infection rate between tourniquet and non-tourniquet groups

Two studies [19,20] demonstrated the postoperative infection rate between the tourniquet (*n* = 66) and non-tourniquet groups (*n* = 68). Heterogeneity was not observed (*P* = 0.88, *I*^2^ = 0%), and the postoperative infection rate was not found to be significantly different between the two groups (RR 1.83, 95% CI (0.65, 5.12)) using the fixed effects model. The finding demonstrates that there is no difference between the tourniquet and non-tourniquet groups with regard to postoperative infection rate (see Figure 5).

**Figure 5:** Meta-analysis of postoperative infection rate in the tourniquet and non-tourniquet groups.

### Comparison of deep venous thrombosis incidence between tourniquet and non-tourniquet groups

Two studies [19,20] reported 134 patients’ deep venous thrombosis state, including 66 in the tourniquet group and 68 in the non-tourniquet group. Heterogeneity was not observed (*P* = 0.84, *I*^2^ = 0%) and the fixed effects model was chosen. Comparison of deep venous thrombosis incidence showed that the tourniquet and non-tourniquet groups were no significantly different (RR 4.13, 95% CI (0.47, 36.17)) under the fixed effects model when homogeneity was found (*P* = 0.84, *I*^*2*^ = 0%) (Figure 6).

**Figure 6:** Meta-analysis of deep venous thrombosis incidence in the tourniquet and non-tourniquet groups.

## Discussion

There is controversy regarding the use of a tourniquet, and the benefits must be weighed against the potential risks. In our meta-analysis, three citations were recruited, all of which were small sample size studies. Tourniquets are used routinely to maintain blood loss during operations on limbs. In this paper, we compared applying and not applying a tourniquet in ankle trauma surgery on operation time, hospital stays, postoperative range of motion, infection rate, and incidence of deep venous thrombosis. Meta-analysis demonstrated no significant differences were observed in operation time, postoperative infection rate, and deep venous thrombosis incidence (*P* >0.05), while significant differences were observed in hospital stays and range of motion (*P* <0.05).

In the previous meta-analysis study, Tai et al. demonstrated that the operation time of knee arthroplasty was significantly shorter in the tourniquet group compared with the non-tourniquet group. In addition, the incidence of clinical thromboembolic events was higher in patients with a tourniquet than those without it [17]. However, Smith et al. stated that the incidence of wound infection and deep vein thrombosis was greater in the tourniquet group than that in the non-tourniquet group, and there was no significant difference in operation time between these two groups [18]. In our study, there were no significant differences between the two groups on the operation time, wound infection, and incidence of deep vein thrombosis, which suggest that larger primary studies are needed for the evaluation of tourniquet efficacy.

Moreover, length of stay is an important outcome as a marker for resource consumption, and prolonged hospital stay can allow insight into the process of postoperative care for patients treated with a tourniquet [22]. In our meta-analysis, tourniquet use was found to extend hospital stay, which further confirms that postoperative care is extremely important for patients with tourniquets. The results were consistent with Smith’s previous study: hospital length of stay was shorter in the non-tourniquet group compared with the tourniquet group during foot and ankle surgery [18]. However, longer hospital stay increased healthcare costs and patients’ burden, and it has been reported that large errors occurred in hospital which suggests a longer stay would not be beneficial for patients’ recovery [23-25]. Additionally, ankle range of motion was significantly decreased in the tourniquet group rather than the non-tourniquet group. Similar to numerous studies [16,26], the use of a tourniquet can restrict joint range of motion due to the excessive tourniquet pressure on the underlying muscle of affected area. In Smith’s study, there was no difference of joint range of motion between the tourniquet and non-tourniquet groups [18].

Some studies [6,27] also reported muscle weakness and nerve injury led by tourniquets in limb trauma surgery, especially in lower limbs, which were not included in the three trials selected in our meta-analysis. Additionally, some papers [28,29] reported that the location of tourniquets might affect postoperative effects. Moreover, other important outcomes such as surgical visualization and technical difficulties during surgery were not assessed in our study. Therefore, all these additional factors should be evaluated in the future study.

Some limitations in our meta-analysis should be acknowledged. First, the number of trials is so small that they may not be adequate to detect the difference between the tourniquet and non-tourniquet groups. Second, funnel plot analysis should be used to assess selection bias. According to the Cochrane handbook for systematic reviews, tests for funnel plot asymmetry should be applied only if there are at least 10 studies included in the meta-analysis [30]. Third, there were methodological flaws in all three trials, such as unclear stochastic method and blind method. Hence, we will select a larger number of trials and use the funnel plot to measure the selection bias in the near future.

## Conclusions

The clinic use of a tourniquet would extend hospital stays and limit patients’ range of motion. No statistically significant differences in operation time, postoperative infection rate, and incidence of deep venous thrombosis were observed between the tourniquet and non-tourniquet groups. However, the evidence base had methodological limitations, most notably in the use of small numbers of trials. Further studies are still required to improve the quality of the evidence base, to determine whether tourniquets should be used on ankle trauma surgery.

## Abbreviations

CI: Confidence intervals; MD: Mean difference; RR: Relative risk; SD: Standardized deviation.

## Competing interests

The authors declare that they have no competing interests.

## Authors’ contributions

XHJ designed research; BQY performed research; WQ contributed analytic tool and analyzed data; JWH wrote the paper. All authors read and approved the final manuscript.
